# Effects of Low-Level Laser Therapy on Osseous Defects Distal to Mandibular Second Molar after Extraction of Impacted Third Molar

**DOI:** 10.1155/2022/9900146

**Published:** 2022-04-21

**Authors:** Ling-Yu Li, Jie Chen, Ming Yu, Yue-Ling Li, Gang Zhou

**Affiliations:** ^1^Dental Comprehensive Department, The Dental Center, Jiading District, Shanghai, China; ^2^Oral and Maxillofacial Surgery, The Dental Center, Jiading District, Shanghai, China

## Abstract

**Objective:**

To evaluate the efficiency of low-level laser therapy on the distal osseous defects of the mandibular second molar (M2) after the adjacent impacted third molar (M3) extraction.

**Methods:**

A total of 59 clinic cases were screened out, whose M3 were impacted and the distal alveolar bone of M2 had been destroyed horizontally. They were randomly divided into 2 groups based on whether they would have laser irradiation or not after M3 extraction. Then, postoperative complications of the 2 groups were compared. The alveolar bone level distal to M2 was established before and 3 to 6 months after M3 extraction by radiographic evaluation, which was compared between two groups.

**Results:**

The incidence of severe pain and mouth-opening limitation was significantly lower in the LLLT group than that in the control group. The amount of bone formation in the LLLT group was higher than that in the control group 3 months after the operation, and the difference was statistically significant. But the difference was not statistically significant 6 months after surgery.

**Conclusion:**

LLLT may alleviate postoperative complications and improve early osteogenesis. It is a viable option for use in the treatment of osseous defects distal to mandibular second molars following extraction of impacted third molars.

## 1. Introduction

The mandibular wisdom teeth, as the latest permanent teeth to erupt in the mandible, often fail to erupt into their normal position due to lack of space in the mandibular arch and soft tissue coverage, with an incidence of 66% to 77% [1]. This can lead to significant resorption of the adjacent second molar distal to the alveolar bone, combined with caries and periodontal disease caused by poor self-cleaning, often resulting in loosening or even extraction of the second molar [2, 3].

Some foreign scholars believe that the distal and middle alveolar bone defect of the second molar can be repaired to a certain extent after the extraction of the impacted wisdom teeth before the age of 25 [4]. Some scholars advocate that artificial bone material and coating barrier membrane should be implanted after the extraction of the mandibular impacted wisdom teeth [5], and platelet-rich plasma (PRP) should be implanted to increase the recovery of alveolar bone tissue of the second molar [6]. However, the results are still controversial, the cost is high, and clinical promotion is difficult.

The new technology of low-energy ultrashort-pulsed electron beam (UPEB) accelerators has been developed opening new directions for radiobiology and biomedical research. Low-energy laser has been proved to have anti-inflammatory and anti-infective effects, accelerating the repair of damaged tissues, and analgesic effects [7–9]. One of the advantages is that these electron accelerators can deliver a very high-peak radiation dose with a low beam charge, thus providing ultrashort dose delivery times. In this study, whether low-energy laser therapy can reduce the postoperative symptoms of mandibular impacted wisdom tooth extraction and promote the formation of adjacent second molar distal alveolar bone were studied.

## 2. Material and Methods

### 2.1. General Information

The subjects were 59 cases of low mesial or horizontal impacted mandibular third molars admitted to Jiading District of Shanghai from November 2018 to November 2020.

### 2.2. Inclusion Criteria

The inclusion criteria are as follows: (1) no tooth extraction contraindications; (2) young, aged 25-35, because most people with M3 extraction are at this age; (3) low mesial or horizontally impacted mandible; and (4) excellent compliance.

### 2.3. Exclusion Criteria

The exclusion criteria are as follows: (1) doubts about the treatment plan or have significant mental and psychological disorders; (2) obvious periodontal disease, caries in the distal root surface of the adjacent wisdom teeth, and alveolar nerve canal compression under the wisdom teeth; (3) followed up less than three times after treatment; and (4) tooth extraction time more than 30 min, because more than 30 minutes might cause damage to the tooth.

## 3. Research Method

### 3.1. Preoperative Test

Understand the medical history and the patients' general condition, improve the preoperative examination (curved slice, laboratory examination, etc.), formulate the operation plan, and sign the informed consent of the operation. According to the random number table method, they were divided into two groups: the experimental group (30 cases were treated with low-energy laser irradiation for 30 minutes) and the control group (29 cases were not treated with low-energy laser irradiation for 30 minutes). Patients were blinded to randomized group assignment. All patients are randomly subjected to treatment or control groups. Randomization can mitigate the biases with randomness.

### 3.2. Surgical Method

(1) Two groups of patients under inferior alveolar nerve block + local infiltration anesthesia, using mandibular second molar distal and buccal angle incision (try not to cut or as far as possible not involved in the vestibular groove), flap to the periosteum, fully exposed the mandibular impacted teeth and surrounding alveolar bone. Remove the crown and bone resistance with a high-speed gas turbine contra-angle dental handpiece, minimally invasive tooth extraction and extraction of root using clavis, scratch the alveolar fossa and saline irrigation, reset the alveolar bone, gelatin sponge gel filling, tension-free suture gingival incision. The stitches are removed on the 7th postoperative day. Postoperative oral antibiotics for 3 days to prevent infection. (2) The experimental group, the Nd-YAG laser (Fotona M021-3AF/3) with a wavelength of 1064 nm was used immediately after the operation in the intraoral surgical area and extraoral temporomandibular area, with a power of 300 NW, an energy density of 3 J/cm2, and irradiation time of 5 min; the control group, the machine was not switched on during the operation and no laser output.

### 3.3. Observation Indicators and Evaluation Criteria

(1) Postoperative pain: stitches were removed on the seventh postoperative day, postoperative cheek pain was assessed by numerical rating scale (NRS) (0 painless, 1-3 mild pain did not affect sleep, 4-6 moderate pain affected sleep, and 7-10 severe pain seriously affected sleep); (2) Mouth-opening degree: on the 7th day after the operation, the patients were followed up to remove the suture and asked and recorded the opening degree when the swelling was most obvious (opening degree 1 and below, opening degree 2, and opening degree 3 and above); (3) Preoperatively: 3 months; postoperatively: 3months and 6 months. The vertical distance *d* (mm) from the distal alveolar crest of adjacent M2 to the distal enamel bone boundary was measured on the curved section (Figures 1, 2, and 3), respectively. The difference between preoperative and postoperative was the vertical regeneration height *D* of the alveolar bone, namely, alveolar bone regeneration height *D* (postoperative 3 M) = d1 − d2; the height of alveolar bone regeneration *D* (postoperative 6) = d1–d3.

### 3.4. Statistical Analysis

Data processing was completed using the SPSS28.0 statistical package and measurement data were expressed as mean ± standard deviation (*i* ± *S*). Comparisons between experimental and control groups were performed using an independent sample *t*-test with *P* < 0.05 as statistically significant.

## 4. Results

The control group included 29 patients. The test group included 30 patients. There was no significant difference in the preoperative bone loss between the experimental and control groups (*P* = 0.644). The average value of the vertical regeneration height of the alveolar bone at the 3rd after surgery was 3.677 ± 0.5488 mm and 3.200 ± 0.6649 mm, respectively, There were significant statistical differences in the regeneration height between the two groups (*P* = 0.004); The average value of the vertical regeneration height of the alveolar bone at 6 months after surgery was 4.097 ± 0.5449 mm and 3.828 ± 0.5098 mm, respectively. There was no significant statistical difference in the regeneration height between the two groups (*P* = 0.055) (Table 1). It is suggested that a low-energy laser could promote the initial healing and osteogenesis of the wound but had no obvious effect on the long term.

The postoperative pain values in the experimental group were significantly lower than those in the control group (*P* = 0.031) and the degree of the opening was greater than that in the control group (*P* = 0.011). The difference was statistically significant (*P* < 0.05) (Table 2), indicating that low-energy laser therapy was significantly effective in providing analgesia and relieving restricted mouth opening after extraction of the obstructed wisdom teeth.

## 5. Discussion

Low-energy laser (LLL) refers to the after laser irradiation of biological tissue, local tissue temperature is not more than 36.5°C or normal body temperature, wavelength range 600-1100 nm, the output power is less than 500 mW, and energy density 1-20 J/cm2. The corresponding treatment method is called low-level laser therapy (LLLT).

The biological mechanism of LLLT is more complex, and it is currently recognized to change the biological behavior [10] of cells by affecting the mitochondrial respiratory chain or cell membrane calcium channels. It can stimulate the activity of macrophages on fibrin absorption while increasing the number of lymphatic vessels, increasing lymphatic reflux, reducing inflammatory exudation, reducing local swelling [11], regulating nerve function, reducing nerve terminal excitability, and playing analgesia.

Multiple studies have shown that LLLT can stimulate bone tissue metabolism and accelerate fracture healing and repair. The Medalha et al. [12] study found that LLLT can accelerate nascent bone deposition, improve the bone healing process of rat tibial defect by activation of osteogenic factors (e. g., RUNX2); the aged rat osteoporosis model conducted by Zhu [13] et al., LLLT was found to increase bone mineral density and improve the bone structure. It also improves the alkaline phosphatase (ALP) and osteocalcin (OCN) levels in the serum and the number of osteoblasts in the bone marrow; besides, LLLT can also affect cellular RNA and DNA synthesis, promote cell proliferation of [14], release of the growth factors, and promote the collagen synthesis of neovascular growth of [15] as well as of fibrotic tissue cells, thus to accelerate the wound tissue healing.

In this experiment, the early bone formation in the distal mandibular second molars was better than that in the control group, and the postoperative pain and opening limitation caused by swellings were also effectively relieved, which improved the postoperative comfort. There are also limitations of this study. First, the number of patients involved is not so large, which needs more people in further studies. Moreover, we did not explain the mechanism of this study, which made it not so credible.

Most researchers believe that the distal middle periodontal condition of the mandibular second molar is not changed or slightly improved after wisdom tooth extraction, but the recovery is closely related to the age, degree of periodontitis, and bone defect at tooth extraction. It was found that after the extraction of the mandibular impacted wisdom teeth, the M2 distal periodontal bone defect could be gradually recovered in those younger than 25 years old, but for those older than 25 years old, the periodontal bone defect in the M2 distance was gradually worsened [16]. In addition, periodontitis itself will lead to the destruction and absorption of the alveolar bone around the teeth, and the uncontrolled bone defect is difficult to recover. The third molar obstruction has caused caries in the neck or root surface of the M2 far-middle teeth, due to the bacterial factors of the neck and root surface caries and later filling, the recovery of periodontal bone tissue is also bound to be affected. Therefore, to exclude the influence of other factors on the experimental results, when screening cases, cases under 25 years of age, periodontitis and cervical caries in M2 distal middle teeth were excluded. In addition, cases over 35 years old with age healing ability difference that is too big were also excluded.

## 6. Conclusion

In conclusion, the results of this experiment confirm that LLLT can effectively reduce the postoperative symptoms of impacted wisdom tooth extraction and promote the early recovery of vertical alveolar bone in adjacent second molars. It is a simple operation method and low treatment cost, which is an effective treatment method suitable for clinical promotion.

## Figures and Tables

**Figure 1:** Preoperative data measurements (d1).

**Figure 2:** Data were measured at 3 months after surgery (d2).

**Figure 3:** Data were measured at 6 months after surgery (d3).

**Table 1:** Comparison of bone increment in M2 distal areas at different periods after M3 extraction.

Group	*n*	Preoperative bone loss	Postoperative 3 M bone increment	Postoperative 6 M bone increment
Experimental group	30	6.580 ± 0.5684	3.677 ± 0.5488 mm	4.097 ± 0.5449 mm
Control group	29	6.514 ± 0.5256	3.200 ± 0.6649 mm	3.828 ± 0.5098 mm
*t* value		0.464	3.007	1.957
*P* value		0.644	0.004	0.055

**Table 2:** Comparison of postoperative pain values and opening degree after M3 extraction.

Group	*n*	Postoperative pain values	Postoperative opening degree
Experimental group	30	2.70 ± 0.988	2.60 ± 0.621
Control group	29	3.41 ± 1.4523	2.10 ± 0.817
*t* value		2.214	2.633
*P* value		0.031	0.011

## Data Availability

The data used to support this study are available from the corresponding author upon request.
